# Analysis of LINC01314 and miR-96 Expression in Colorectal Cancer Patients via Tissue Microarray-Based Fluorescence *In Situ* Hybridization

This article has been retracted.

**DOI:** 10.1155/2022/5378963

**Published:** 2022-10-07

**Authors:** Runan Zhang, Genhua Zhang, Baohua Li, Juan Wang, Jvfang Wang, Jia Che, Xiaojun Wang, Zhen Zhang

**Affiliations:** ^1^Department of Clinical Laboratory, Tongde Hospital of Zhejiang Province, Hangzhou, Zhejiang, China; ^2^Department of Pathology, Tongde Hospital of Zhejiang Province, Hangzhou, Zhejiang, China

## Abstract

**Methods:**

A tissue microarray (TMA) containing 76 individual colorectal tumor samples and 28 adjacent normal samples was constructed, and the expression levels of LINC01314 and miR-96 were detected by fluorescence in situ hybridization.

**Results:**

The expression levels of both LINC01314 and miR-96 were upregulated in CRC tissues and were associated with vascular metastasis (*p* < 0.05). A significantly positive correlation was observed between LINC01314 and miR-96 expression in tumor tissues (*p* < 0.001, *r* = 0.870). Dominant expression of LINC01314 was a risk factor for both blood vessel invasion (*p* < 0.05) and poor 5-year survival (*p* = 0.001, hazard ratio = 4.144). The Kaplan–Meier analysis indicated that patients with LINC01314-dominant expression exhibited worse 5-year survival rates than those with miR-96-dominant expression (*p* < 0.05).

**Conclusion:**

The expression patterns of both LINC01314 and miR-96 may be diagnostic of, and prognostic for, CRC. These findings will facilitate further exploration of the molecular mechanism of lncRNAs in CRC.

## 1. Introduction

Colorectal cancer (CRC) is the second most common cause of cancer mortality worldwide, with more than 1.93 million diagnoses and 930,000 deaths annually (World Cancer Report 2020) [1]. In China, 550,000 cases and 280,000 deaths are reported each year [2]. Early CRC is curable, and the tumors can be removed surgically. Unfortunately, CRC is often advanced when diagnosed, associated with distant metastases [3]. Biomarkers that detect early cancer and/or predict prognosis have been extensively studied [4–6]. However, 5-year survival remains poor; CRC pathogenesis is not well-understood. Novel biomarkers facilitating early diagnosis, prognostic predictions, and treatment are urgently required.

Long noncoding RNAs (lncRNAs) have recently attracted attention as biomarkers for CRC diagnosis and prognostication [7]. lncRNAs (>200 nucleotides in length) are widespread in many species [8]. Accumulating evidence suggests that lncRNAs engage in transcriptional regulation (thus gene-specific transcription) and posttranscriptional and epigenetic regulation [9, 10]. Several lncRNAs are aberrantly expressed in various cancers and function as tumor suppressors, promoters, or both under certain conditions by combining with proteins or nucleotide sequences to regulate downstream molecules [11–15]. For example, growth arrest specific 5 (GAS5) and LINC01559 exhibit antioncogenic effects in CRC development or progression. Low-level expression of lncRNA GAS5 and/or LINC01559 is associated with a poor prognosis in CRC patients [16, 17]. Meanwhile, HOX transcript antisense RNA (HOTAIR) and colon cancer-associated transcript 1 (CCAT1) were found to be upregulated in the early stages of colorectal carcinogenesis and associated with TNM stage and poor overall survival [18–20]. Similarly, LINC01314 was demonstrated to repress gastric cancer progression by modulating Wnt/*β*-catenin signaling [21]. Lv et al. reported that LINC01314 overexpression reduced hepatoblastoma cell proliferation and migration [22]. However, few reports have explored the expression levels, molecular effects, and clinical significance of LINC01314 in CRC patients.

MicroRNAs (miRNAs) are single-stranded noncoding RNAs that regulate gene expression via base-pairing. Interactions between lncRNAs and miRNAs regulate several biological and pathological processes [23–25]. The molecular details of lncRNA–miRNA crosstalk in terms of CRC progression were summarized by Wang et al. [26]. TargetScan revealed that LINC01314 shared a binding site with miR-96; the molecules may interact. We thus explored LINC01314 and miR-96 expressions in CRC patients via tissue microarray- (TMA-) based fluorescence in situ hybridization (FISH). We speculated that LINC01314 and miR-96 expression patterns might be both diagnostic of, and prognostic for, CRC.

## 2. Materials and Methods

### 2.1. Specimens and Clinical Data

Tumor tissues and adjacent normal tissues were obtained from patients who underwent surgery to treat primary CRCs in the Tongde Hospital of Zhejiang Province (People's Republic of China) in 2015 and 2016. All specimens were independently diagnosed histologically by three experienced pathologists by reference to the NCCN Clinical Practice Guidelines in Oncology for Colon Cancer (ver. 3, 2013) [27]. Residual tissues were immediately frozen in liquid nitrogen. The study was approved by the Ethics Committee of Tongde Hospital, Zhejiang Province (reference number: 2021025). All patients provided written informed consent in accordance with the 1975 Declaration of Helsinki. Patients were followed-up every 6 months for 5 years after primary surgery; survival, the dates of any events, and the causes of death were recorded. The median overall survival was 48 months, and the patient age ranged from 34 to 95 years (median 70 years). Clinicopathological data (tumor size; pathological pattern; blood vessel invasion, lymph node metastasis, and nerve invasion statuses; and TNM stage) were retrieved from pathology reports lodged in the hospital information system. The clinical and pathological characteristics of 76 CRC patients are listed in Table 1.

### 2.2. TMA Analysis

A colorectal TMA was constructed as described previously [28–30]. Briefly, tumor and adjacent normal tissues were fixed in 4% (*v*/*v*) formalin and embedded in paraffin. Donor blocks were subjected to hematoxylin and eosin (H&E) staining to identify representative tumor regions. Tissue cylinders (6 mm diameter) were punched from target areas and inserted into recipient paraffin blocks using an automatic precision instrument. Each TMA block featured 76 individual colorectal tumor samples and 28 adjacent normal samples. Each TMA block was then cut into several 4 *μ*m thick sections (HistoCore BIOCUT, Leica, Wetzlar, Germany), and the sections were mounted on glass slides for H&E staining and FISH.

### 2.3. FISH

LINC01314 and miR-96 in TMA samples were detected via FISH, as described previously [16, 31–33]. After deparaffinization and air-drying, TMA slides were immersed in DEPC-treated RNase-free water and incubated in 0.01 M citric acid buffer (pH 6.0) at 95°C for 10 min, followed by proteinase K digestion for 20 min. After prehybridization for 1 h, slides were incubated with a 1 *μ*M solution of the Spectrum-CY3-labeled miR-96 probe (5′-CY3-GCAAAAATGTGCTAGTGCCAAA-CY3-3′) and the Spectrum-FAM-labeled LINC01314 probe (5′-FAM-GGTGGATGTGGGGATGGCGCTGTAAGGG-FAM-3′) in hybridization buffer overnight at 42°C in a humidified chamber. The slides were washed in graded SCC solutions (2×, 1×, and 0.5× SCC for 10 min each), and the nuclei were counterstained with 4′,6-diamidino-2-phenylindole (DAPI; Cell Signaling Technology, Danvers, MA, USA) for 8 min. Images were obtained using a fluromicroscope (Nikon ECLIPSE C1, Tokyo, Japan) at 100x magnification.

### 2.4. Statistical Analysis

Statistical analysis was performed using SPSS ver. 26.0 (IBM Corp., Armonk, NY, USA) and GraphPad Prism ver. 9.0 (GraphPad Software, San Diego, CA, USA). LINC01314 and miR-96 levels in tumor tissues were subjected to the Pearson correlation analysis. Associations between LINC01314 and miR-96 expressions and pathological characteristics were evaluated using Student's *t*-test and ANOVA. Possible risk factors for tumor vascular invasion and 5-year mortality were explored using logistic regression and Cox's regression analyses. The survival rates of the LINC01314- and miR-96-dominant groups were compared using the Kaplan–Meier method. A *p* value *<* 0.05 was considered significant.

## 3. Results

### 3.1. Expression of LINC01314 and miR-96 as Revealed by TMA-Based FISH

TMA blocks containing 76 and 28 tumor and normal tissue samples, respectively, were constructed. A complete H&E-stained block is shown in Figure 1(a). One H&E-stained TMA spot is shown in Figures 1(b) and 1(c). FISH was used to detect LINC01314 and miR-96 expressions (Figure 2). Representative TMA sections exhibiting LINC01314 and miR-96 expressions are shown in Figure 3. The extent of RNA expression was measured by recording the integrated optical density (IOD) using ImageJ software. As normal tissue sections barely fluoresced, data were compared based on the relative IODs (IOD of tumor tissues divided by the mean IOD of normal tissues). The mean relative IODs of LINC01314 and miR-96 were significantly higher in tumor tissues than normal tissues (77.3 ± 232.1 vs. 1 and 31.2 ± 62.5 vs. 1, respectively; data not shown). A significantly positive correlation was observed between LINC01314 and miR-96 expressions in tumor tissues (*p* < 0.001, *r* = 0.870, Figure 4).

### 3.2. Clinical Significance of LINC01314 and miR-96 Expressions in CRC Patients

Tissue samples were divided into several groups according to the clinicopathological characteristics, and LINC01314 and miR-96 expression levels were compared. In contrast to the vascular nonmetastasis group, tissues in the metastasis group expressed significantly lower levels of LINC01314 (21.89 ± 39.178 vs. 109.15 ± 284.897, *p* < 0.05) and miR-96 (10.30 ± 15.292 vs. 43.98 ± 75.010, *p* < 0.05, Table 1). ANOVA revealed that LINC01314 expression was associated with tumor invasion depth (*p* < 0.05, data not shown) and miR-96 expression was associated with tumor differentiation (*p* < 0.05). However, neither expression level differed by age, sex, tumor size, histological type, TNM stage, lymph node metastasis status, nerve invasion, or survival.

### 3.3. LINC01314-Dominant Expression Is a Risk Factor for Tumor Vascular Metastasis and Poor 5-Year Survival

To further analyze the relationships of LINC01314 and miR-96 expressions with the clinical characteristics of CRC patients, we introduced the concept of dominant expression. If the relative IOD of LINC01314 was higher than that of miR-96 in a TMA section, the patient was considered to exhibit LINC01314-dominant expression and vice versa. Of the 76 CRC patients, 52 exhibited LINC01314-dominant expression and 24 miR-96-dominant expression. Potential risk factors for tumor vascular metastasis (age, sex, tumor size, tumor location, histological type, extent of differentiation, TNM grade, nerve invasion, and LINC01314-dominant expression) were evaluated via logistic regression analysis. As shown in Table 2, tumor vascular metastasis was significantly associated with both the TNM grade and LINC01314-dominant expression (*p* = 0.003 and *p* = 0.029, respectively). Cox's regression analysis indicated that age (*p* = 0.029, hazard ratio (HR) = 1.029), TNM grade (*p* = 0.015, HR = 0.470), and LINC01314-dominant expression (*p* = 0.001, HR = 4.144) were significantly associated with poor 5-year survival (Table 3). Thus, LINC01314-dominant expression is a risk factor for both tumor vascular metastasis and poor 5-year survival in CRC patients.

### 3.4. LINC01314-Dominant Expression Was Associated with Poor 5-Year Overall Survival

The mean survival time of the 76 CRC patients was 44.2 ± 17.1 months (range 12–60 months); 44.2% (23/52) of patients with LINC01314-dominant expression remained alive during follow-up. The 5-year survival rate of the patients with miR-96-dominant expression was 54.2% (13/24). The Kaplan–Meier analysis indicated a significant difference in survival curves between the two groups of patients (*p* = 0.048). As shown in Figure 5, patients with LINC01314-dominant expression exhibited worse 5-year survival rates.

## 4. Discussion

CRC is one of the most frequently diagnosed cancers worldwide, including China, and over 80% cases are initially diagnosed at an advanced stage [34]. It is critical to develop indicators aiding diagnosis and/or predicting prognosis. We are the first to simultaneously evaluate LINC01314 and miR-96 expressions in CRC TMA blocks via FISH and to explore the correlations between expression patterns and clinicopathological characteristics. Both LINC01314 and miR-96 expression levels were significantly higher in tumor tissues and were associated with vascular metastasis. Cox's regression analysis showed that LINC01314-dominant expression was associated with an increased risk of death in CRC patients. LINC01314 and miR-96 expression patterns will aid the diagnosis and/or prognosis of CRC patients.

miR-96 is involved in many critical cellular processes including proliferation, differentiation, and apoptosis [23, 35]. However, the role played by miR-96 in colorectal carcinogenesis remains unclear. Yue et al. reported that miR-96 triggers CRC development and progression via the AMPK*α*2-FTO-m6A/MYC axis [36]. Ress et al. suggested that lower miR-96 values were associated with metastases and shorter survival in CRC patients [37]. In vitro, overexpression of miR-96 reduced cellular growth as reflected by increased p27-CDKN1A and decreased cyclin D1 expression [37]. We found that miR-96 was expressed more highly in tumor than normal tissues and that lower expression was associated with vessel invasion, consistent with the Ress data. The Cancer Genome Atlas RNA-seq data show that LINC01314 is aberrantly expressed in various tumors, showing upregulation in thyroid carcinoma but downregulation in cholangiocarcinoma, esophageal carcinoma, kidney chromophobes, kidney renal papillary cell carcinoma, kidney carcinoma, lung adenocarcinoma, pheochromocytoma, and paraganglioma [12]. However, LINC01314 expression and function in CRC have not been investigated. We found that LINC01314 expression was higher in CRC tissues than normal tissues and that lower expression was associated with tumor invasion. These results improve our understanding of the role played by LINC01314 during colorectal carcinogenesis.

The lncRNA–miRNA–mRNA axis is a novel regulatory mechanism featuring interactions among lncRNAs, miRNAs, and mRNAs, and it plays a crucial role in the pathophysiological steps of tumor carcinogenesis, progression, and metastasis [38–41]. Most CRC-related lncRNAs have been reported to be upregulated and appear to function as miRNA sponges [7]. lncRNAs are involved in a variety of tumor-related pathways, such as the estimated growth factor receptor (EGFR), Wnt, and p53 signaling pathways, by regulating miRNAs [41]. For example, nuclear-enriched abundant transcript 1 (NEAT1) promoted CRC tumorigenesis through various lncRNA/miRNA axes, such as the NEAT1/miR-495-3P/CDK6 [42], NEAT1/miR-34a/SIRT1/Wnt/-catenin [43], and NEAT1/miR-205-5p/VEGFA axes [44]. In the present study, LINC01314 and miR-96 expression levels were found to be positively correlated in CRC tumor tissues, and both were associated with vessel invasion. Bioinformatics analysis suggested that a binding site is shared by LINC01314 and miR-96. We suggest that LINC01314–miR96 is a novel epigenetic regulatory axis involved in CRC development. More importantly, LINC01314-dominant expression was associated with higher risks of vessel invasion and poorer survival compared with miR-96-dominant expression in CRC patients. We speculate that LINC01314 may promote the development of CRC by reducing the ability of miR-96 to slow tumor progression, thereby reducing the survival of CRC patients. These speculations and the underlying crosstalk mechanisms between LINC01314 and miR-96 in CRC development will be demonstrated in our future *in vitro* experiments.

N6-methyladenosine (m6A) modification is among the most ubiquitous epigenetic modifications of mRNAs and noncoding RNAs (e.g., miRNAs and lncRNAs) [45]. Overwhelming evidence indicates that the dysregulation of m6A modification is significantly correlated with CRC tumorigenesis and progression [46, 47]. lncRNAs and miRNAs are not only important targets of m6A modification regulators; they also regulate m6A modification [48, 49]. Whether LINC01314 and miR-96 affect the development of CRC carcinogenesis through m6A methylation modification remains to be explored in a future study.

LINC01314 and miR-96 expressions were detected via TMA-based FISH, which affords many advantages compared with traditional methods. Aggregation of many tissues and experimentation under identical conditions optimize standardization [50]. A single tumor block can be cut into many sections, and repeat evaluations are possible. However, there were two major limitations that we plan to address. First, any retrospective study is associated with a risk of selection bias. Second, the interactions between LINC01314 and miR-96 and their roles in CRC progression must be investigated in vitro. We will establish a prognostic CRC model featuring lncRNA and miRNA detection and perform a large, prospective cohort study. This research will improve our understanding of the molecular mechanism of lncRNAs and miRNAs in CRC development and provide a novel strategy for the clinical diagnosis and prognosis of CRC.

## 5. Conclusion

In conclusion, we found that LINC01314 and miR-96 expression levels were upregulated in CRC tissues and were associated with vascular metastasis. LINC01314-dominant expression was a risk factor for tumor vascular invasion and poor 5-year survival in CRC patients. LINC01314 and miR-96 may be used as novel biomarkers for the diagnosis, prognostic predictions, and treatment of CRC. Combined detection of the expression of LINC01314 and miR-96 in tumor tissues and expression pattern analyses will aid CRC diagnosis and prognosis.

## Figures and Tables

**Figure 1:** Colorectal cancer (CRC) tissue microarray (TMA). (a) Hematoxylin and eosin- (H&E-) stained complete TMA containing 76 individual tumor samples and 28 adjacent normal tissue samples. The arrangement of the TMA template is shown in Supplementary Figure 1. (b) H&E-stained normal tissue. (c) H&E-stained CRC tumor tissue.

**Figure 2:** Complete TMA scan under fluorescence microscopy obtained following fluorescence *in situ* hybridization (FISH) analysis. Nuclei were stained with 4′,6-diamidino-2-phenylindole (DAPI; blue). The arrangement of the TMA template is consistent with the H&E-stained TMA in Supplementary Figure 1.

**Figure 3:** Representative TMA sections exhibiting low, medium, and high LINC01314 or miR-96 expression. After hybridization, images were obtained using a fluromicroscope at 100x magnification. Tumor tissues expressed LINC01314 and miR-96 to varying degrees; representative images are shown. miR-96 showed red fluorescence (above), LINC01314 showed green fluorescence (below), and nuclei showed blue fluorescence.

**Figure 4:** Correlation between LINC01314 and miR-96 expressions analyzed by the Pearson correlation analysis. LINC01314 and miR-96 expressions in each tumor sample are presented in the coordinate system. Dots represent individual colon tumor samples. A significantly positive correlation was observed between LINC01314 and miR-96 expressions in tumor tissues (*p* < 0.001, *r* = 0.870).

**Figure 5:** Comparison of 5-year overall patient survival between the LINC01314-dominant expression (dashed line, 44.2%) and miR-96-dominant expression (solid line, 54.2%) groups, analyzed using the Kaplan–Meier method. Patients with LINC01314-dominant expression exhibited worse 5-year survival rates than those with miR-96-dominant expression (*p* = 0.048).

**Table 1:** Clinical data of the 76 CRC patients.

Clinical characteristics	*n*	Relative LINC01314 expression (mean ± SE)	*p* value	Relative miR-96 expression (mean ± SE)	*p* value
Age (years)^a^					
<60	10	38.90 ± 83.594	0.573	24.50 ± 50.131	0.718
≥60	66	83.71 ± 247.045		32.25 ± 64.450	
Gender^a^					
Male	36	82.11 ± 134.726	0.880	38.71 ± 65.954	0.334
Female	40	73.90 ± 293.864		24.65 ± 60.308	
Tumor size (cm)^a^					
<5	32	99.81 ± 327.512	0.481	28.59 ± 62.231	0.756
≥5	44	61.30 ± 122.852		33.16 ± 63.349	
TNM stage^a^					
I+II	41	96.32 ± 299.574	0.450	33.83 ± 72.156	0.693
II+IV	35	55.32 ± 105.207		28.06 ± 49.269	
Lymph node metastasis^a^					
Yes	35	55.32 ± 105.207	0.450	33.83 ± 72.156	0.693
No	41	96.32 ± 299.574		28.06 ± 49.269	
Nerve invasion^a^					
Yes	29	53.34 ± 107.095	0.474	25.10 ± 46.795	0.505
No	47	93.11 ± 284.293		35.07 ± 70.853	
Vascular metastasis^a^					
Yes	27	21.89 ± 39.178	0.042	10.30 ± 15.292	0.005
No	49	109.15 ± 284.897		42.98 ± 75.010	
Differentiation^b^					
Poorly	15				
Moderately	58		0.363		0.037
Highly	3				
Histological type^b^					
Ulcerative type	37				
Fungating type	36		0.208		0.212
Infiltrating type	3				

Abbreviations: SE: standard error. ^a^Differences were compared by using Student's *t*-test. Data were presented as the mean ± SE. ^b^Differences were compared by using ANOVA test.

**Table 2:** Logistic regression analyses of risk factors for vascular metastasis.

Variables	*p* value	OR	95% CI
Age	0.588	0.970	0.867-1.084
Gender	0.554	0.499	0.050-4.988
Tumor size	0.879	1.192	0.124-11.472
Nerve invasion	0.240	4.409	0.372-52.279
Lymph node metastasis	0.003	699.227	9.982-48980.134
LINC01314-dominant expression	0.029	611.880	1.900-197023.031
Differentiation	0.975	/	/
Histological type	0.580	/	/
Tumor location	0.960	/	/

Abbreviations: OR: odds ratio; CI: confidence interval.

**Table 3:** Cox's regression analyses for overall survival.

Variables	*p* value	OR	95% CI
Age	0.029	1.029	1.003-1.056
TNM stage	0.016	0.407	0.225-0.868
LINC01314-dominant expression	0.001	4.144	1.823-9.423

Abbreviations: TNM: tumor/node/metastasis; OR: odds ratio; CI: confidence interval.

## Data Availability

The data used in this research are available from the corresponding author upon reasonable request.

## Supplementary Materials

Supplementary Materials Supplementary 1: the arrangement of TMA template.
